# The Influence of Martial Arts on Spine CT Image Morphological Structure Based on Optimized Ant Colony Algorithm

**DOI:** 10.1155/2022/2725819

**Published:** 2022-08-23

**Authors:** Hou Yuhuan, Hou Xueting, Wang Weiyue

**Affiliations:** ^1^Basic Medicine Department, Hubei College of Chinese Medicine, Jinzhou, Hubei 434000, China; ^2^Dankook University College of Physical Education, Yongin, Gyeonggi Province 330712, Republic of Korea; ^3^College of Life Sciences, Guangxi Normal University, Guilin, Guangxi 541000, China; ^4^Shenyang Sports Universitye, Shenyang, Liaoning 110102, China; ^5^Wuhan Sports University, Wuhan, Hubei 430079, China

## Abstract

As the second lifeline of human body, the abnormal development of its morphological structure has a great impact on people's physical and mental health. Due to bad living habits and learning pressure, the morphological and structural development of spine in adolescents and children is abnormal to a certain extent, which can be improved by sports intervention. Therefore, this article puts forward the research on the influence of Wushu on the spinal morphological structure based on the optimization algorithm and integrates the optimization ant colony algorithm on the basis of the traditional spinal CT image segmentation method. The experimental results show that the improved CT image segmentation method based on the optimized ant colony algorithm can solve the sensitive problem of the number of clusters, improve the segmentation efficiency and quality, and provide more accurate data for the subsequent comparative experiments. At the same time, the comparative test results show that Wuqinxi Wushu can better improve the abnormal dry tilt angle, abnormal kyphosis angle, and body balance angle of teenagers, improve the activity of teenagers' spine, and help teenagers enhance the overall health of spine.

## 1. Introduction

Spine is the second lifeline of human body, and its abnormal development has a negative impact on human life. The key period of spinal development is in human adolescence, which is also the golden period of physical development of adolescents and children. With the growth of age, the height and weight of teenagers will continue to increase. If there are nutritional imbalance and lack of exercise at this time, coupled with the low content of inorganic salts in the bones of teenagers and children, under the condition of relatively low bone hardness, teenagers' spine is easy to be deformed under the influence of bad living habits or gravity compression of the external environment, resulting in abnormal spine development [1]. With the development of information technology, while the academic pressure of teenagers has been increasing in recent years, the homework and curriculum tasks completed through the information network are also increasing. Many teenagers' spine has been deformed due to long-time desk writing, poor sitting posture, long-term bow, and heavy schoolbag pressure, even some teenagers and children have spinal lesions, and the prevalence of spine is increasing every year [2]. Therefore, scientific and effective intervention research on spinal development of adolescents and children has become a hot spot in the society.

In the past, relevant experts focused more on the abnormal spinal morphology of adults and the elderly and paid less attention to the abnormal spinal morphology and structure of adolescents and children [3]. However, with the increasing incidence rate of spine and younger age of onset, the spine research is deepening and attention is being paid to the development of spinal column in young children. According to relevant research experience, sports is the simplest means to correct spine shape. Some scholars use Yoga treatment to treat female college students with scoliosis [4]. The quality results show that Yoga treatment has significantly improved scoliosis and shoulder balance, and the mobility of spine in all aspects has also been improved; it shows that Yoga treatment has an effect on spinal correction [5]. Some scholars conducted comprehensive intervention on middle school students with abnormal spinal development for two months, and through the comparison of spinal morphology measurement results before and after the experiment, it is concluded that the degree of spinal abnormality has been greatly reduced, and more than half of the students' spinal posture can return to the normal state, which has a significant improvement effect on spinal abnormality [6]. Other scholars used Taijiquan to treat the middle-aged and elderly patients with lumbar pain symptoms for six months [7]. The chronic low back pain symptoms of the experimental subjects were relieved, and the lumbar spine function was improved [8]. Based on this, some scholars have proposed to effectively intervene the spine morphological development of adolescents and children through martial arts science, so as to help teenagers and children maintain and improve the healthy state of spinal development [9].

However, at present, there is relatively little research on the impact of martial arts on spinal morphological development [10]. Therefore, this paper proposes the impact of martial arts on spinal morphological structure based on the optimized ant colony algorithm [11]. Through the improved CT image segmentation method of the optimized ant colony algorithm, this paper analyzes all aspects of the experimental object's spinal CT images before and after the experiment [12]. This paper is mainly divided into three parts [13]. The first part expounds the influencing factors of spinal morphological structure development and the harm of abnormal development; the second part is the construction of the spine development evaluation model based on optimized ant colony; the third part is the experimental results and analysis of the influence of spine shape and structure of Wushu team based on the optimized ant colony algorithm [14].

The innovation of the research lies in the integration of the optimized ant colony algorithm on the basis of traditional spine CT image segmentation methods. This algorithm can solve the sensitive problem of clustering number, improve the efficiency and quality of segmentation, and provide more accurate data for subsequent comparative experiments. Compared with the traditional fuzzy c-means classification method, the improved CT image segmentation method based on the optimized ant colony algorithm solves the problem of being sensitive to the number of clusters and improves the segmentation efficiency while ensuring the quality of image segmentation. Based on the optimization algorithm, the influence of Wushu on the spine shape and structure was analyzed. It can improve the abnormal development of teenagers' spine and help teenagers improve their overall health.

## 2. Factors Affecting the Development of Spinal Morphology and Structure and the Harm of Abnormal Development

The human spine is located in the middle of the back of the human body and is the backbone of the human body [15]. The spine has a central axial bone structure, which plays a role of lever and supporting weight-bearing in the human body [16]. The physiological bending of the spine can improve the elasticity of the spine and buffer and disperse the gravity and impact on the intracranial central nerve [17]. The flattening of the intervertebral disc in the spine can help the spine to achieve movement and complete complex movements and expand the range of motion of the spine [18]. As can be seen, spine has a very important impact on human activities [19]. Abnormal spinal morphological development has a serious adverse impact on the life and learning of teenagers and children [20].  Figure 1 shows a comprehensive view of the spine.

There are three main influencing factors in the development of spine, namely, genetic factors, lifestyle and habits, and exercise factors [21]. Common spinal diseases such as mandatory spondylitis and adolescent idiopathic scoliosis are affected by genetic genes. Although genetic gene is a very important factor in the development of spine in adolescents and children, it is not a decisive factor. The acquired development of spine is also affected by the living habits and styles of adolescents and children, including positive and negative effects [22]. According to the relevant research results, the quality and manner of teenagers' backpacks will affect the development of their spine morphology, that is, the heavier the backpack is, the more obvious the morphological changes of teenagers' spine will be, which improves the possibility of spine damage [23]. At the same time, teenagers' bad habits such as unilateral backpacking and long-term incorrect sitting posture will increase the burden on the spine, affect the activity and development health of different parts of the spine, and improve the probability of spinal disease. In addition, according to relevant studies, reasonable and appropriate exercise will have a positive impact on the development and morphological structure of teenagers' spine, while different exercise modes and mild exercise have different effects on the spine. Therefore, in the process of helping teenagers and children maintain and improve spinal development and morphological structure, we should find appropriate sport methods.

Abnormal development of spinal morphology and structure will not only bring physical harm to teenagers and children but also have a negative impact on their psychology. According to relevant statistical data, the number of Chinese teenagers suffering from scoliosis of different degrees accounts for 20% of the total number of teenagers and children. More than 80% of teenagers have poor physical posture, of which the most common and serious problem is poor sitting posture, neck probing, and chest hunchback when walking [24]. Such a situation is not only conducive to physical and mental health in the process of teenagers' growth but also has a serious impact on their behavior in future study and life. The abnormal development of spinal morphology and structure is very harmful to the health of adolescents. For example, when the most common scoliosis is in a serious state, it will damage lung function, produce waist and back pain, and affect the biological stress balance of spine [25]. If we cannot take effective measures to intervene and treat in time, it will not only aggravate the condition but also increase the difficulty of treatment.

## 3. Construction of Spine Development Evaluation Model Based on Optimized Ant Colony Algorithm

Due to the gradual aging of the lumbar spine in the middle-aged and elderly, scoliosis can be found in the frontal view. From the lateral position, the disappearance of physiological protrusion may occur, and the disappearance of cervical physiological protrusion may occur in the cervical spine, or spinal deformity is caused by degenerative diseases such as cervical spondylosis. Adolescent spinal deformities, such as scoliosis, can be divided into idiopathic scoliosis, congenital scoliosis, and scoliosis secondary to the muscular nervous system. With the development of science and technology and computer technology, the medical means of analyzing the abnormal development and disease causes of human spine are also constantly developing and updating. Among them, biological realistic model is a method that can present the true state of spine, which integrates computer graphics, digital image processing, medical image knowledge, and other disciplines. It mainly carries out three-dimensional reconstruction of the biological realistic model based on spinal CT images. It is one of the methods to judge the morphological structure of spinal development. Image segmentation is an important part of image 3D reconstruction. The quality of image segmentation is directly related to the accuracy of image analysis, understanding, and 3D reconstruction. Medical image segmentation is to segment the required regions in the image according to the differences between regions and the similarity within regions. At the same time, it should ensure that there is no overlap between the regions of the segmented image. Let all the region sets of the image be represented as *R*, and nonempty region segmented by it be represented as *R*_1_, *R*_2_,…, *R*_*n*_. There are four conditions to be met. The first one is shown in the following formula:

(1) $$\begin{array}{c} R=\cup_{i=1}^{n}R_{i}. \end{array}$$

Second, the two random subregions need to meet the conditions, as shown in the following formula:

(2) $$\begin{array}{c} R_{i}\cap R_{j}=\emptyset , \end{array}$$

in which *i* ≠ *j*. Third, all subregions are nonempty, that is, *R*_*i*_=∅, *i*=1,2,…, *n*; fourth, all subregions are connected regions.

### 3.1. CT Image Segmentation Method Based on Fuzzy C-Means Clustering

Fuzzy C-means clustering method is a clustering algorithm that uses the membership function to determine the clustering degree of pixels. Its core idea is to divide the objects with the greatest similarity into the same cluster, and the similarity between different clusters is the smallest. Let the vector be expressed as *X*_*i*_ and *i*=1,2,…, *n*, and its number is *n*. Divide it into fuzzy subsets with the number of *c* and 2 ≤ *c* ≤ *n*. The membership degree of sample points is expressed as *μ*_*ik*_, and the classification results can be expressed by fuzzy membership degree matrix, as shown in the following formula:

(3) $$\begin{array}{c} U=\left\{\mu_{ik}\right\}, \end{array}$$

in which *μ*_*ik*_ ∈ (0,1). The membership degree is normalized to obtain the following formula:

(4) $$\begin{array}{c} \sum_{i=1}^{c}\mu_{ik}=1, \end{array}$$

in which *k* ∈ [1, *n*].

The value function expression of fuzzy c-means clustering is shown in the following formula:

(5) $$\begin{array}{c} J_{m}\left(U,V:X\right)=\sum_{i=1}^{c}\sum_{k=1}^{n}{\left(\mu_{ik}\right)}^{m}{\left|\left|X_{k}-X_{i}\right|\right|}_{A}^{2}, \end{array}$$

where the strength matrix is expressed as *U*, the positive definite matrix is expressed as *A*, the central point set of clustering fuzzy subset is expressed as *V*=(*v*_1_, *v*_2_,…, *v*_*c*_), and the weighted index is expressed as *m* ∈ [1, *∞*). In order to solve the optimization of formula (5), formula (6) is obtained by constructing Lagrange functional, as follows:

(6) $$\begin{array}{c} \bar{J}\left(U,V:X\right)=J\left(U,V:X\right)+\sum_{j=1}^{n}\lambda_{i}\sum_{i=1}^{c}\left(\mu_{ik}-1\right)=\sum_{i=1}^{c}\sum_{k=1}^{n}{\left(\mu_{ik}\right)}^{m}{\left|\left|X_{k}-X_{i}\right|\right|}_{A}^{2}+\sum_{j=1}^{n}\lambda_{i}\left(\sum_{i=1}^{c}\mu_{ik}-1\right), \end{array}$$

where the Lagrange multiplier is expressed as *λ*_*i*_, *i*=1,2,…, *n*. Calculate the partial derivative of all functional variables used in formula (6) to achieve the minimum necessary condition for realizing the optimal solution, as shown in the following formulas:

(7) $$\begin{array}{c} c_{i}=\frac{\sum_{j=1}^{n}\mu_{ij}^{m}x_{j}}{\sum_{j=1}^{n}\mu_{ij}^{m}}, \end{array}$$

(8) $$\begin{array}{c} \mu_{ij}=\frac{1}{{\sum_{K=1}^{n}\left(d_{ij}/d_{kj}\right)}^{2/\left(m-1\right)}}, \end{array}$$

where the Euclidean distance between the *j* point and the *i* cluster center is expressed as *d*_*ij*_.

### 3.2. Improved CT Image Segmentation Method Based on Optimized Ant Colony Algorithm

The image segmentation by the fuzzy c-means clustering method has good quality and retains the complete information of the required region, but the segmentation time is relatively long. In order to reduce the number of iterations and improve the efficiency of segmentation, this paper introduces the optimal ant colony clustering algorithm.

Ant individuals are very simple social insects, but when they carry out group activities, they can complete extremely complex behaviors through the cooperation between individuals, showing the intelligence in their social tasks. An ant colony can find the shortest path between the nest and food when looking for food and can make corresponding adjustments in a short time when the external environment changes. Ant colony can complete these behaviors, which mainly rely on information hormone, which can transmit the signal to be expressed by individual ants to the latter, so as to affect the behavior of the latter. In addition, if there are obstacles on the way of ant colony foraging, the individual ant choosing the shortest path will release information hormone and affect the behavior of the following ants. With the higher content of information hormone, as shown in Figure 2.

The optimized ant colony image segmentation algorithm mainly includes the characteristics of systematicity, distributed computing, self-organization, and positive feedback. As shown in Figure 3, it is an improved CT image segmentation flow chart integrating the optimized ant colony algorithm. The ant colony clustering algorithm is used to extract the initial cluster center of the image to be segmented, and then the fuzzy c-means algorithm is used to segment the image based on the initial cluster center.

Let the image be expressed as *X*, the pixel *X*_*i*_ in the image is regarded as an ant individual, and each ant has three directional vectors of gradient, gray, and domain features. The distance between the pixel and the cluster center is expressed as *d*_*ij*_, which is calculated by Euclidean distance, as shown in the following formula:

(9) $$\begin{array}{c} d_{ij}=\sqrt{\sum_{k=1}^{m}p_{k}{\left(X_{ik}-C_{jk}\right)}^{2}}. \end{array}$$

The basic characteristic dimensions of ants are *m* and *m*=3, and the weighted silver of each dimension is *p*_*k*_.

The amount of information contained in the area is expressed as *ph*_*ij*_, the influence range of ant individuals on the amount of information in the surrounding local area is expressed as *r*, and the influence degree is shown in the following formula:

(10) $$\begin{array}{c} ph_{ij}=\left\{\begin{array}{c} 1,d_{ij}\leq r;\\ 0,otherwise. \end{array}\right. \end{array}$$

When the ant individual makes path selection, let the attraction factor from the current pixel to the cluster center at the *t* iteration be expressed as *p*_*ij*_^*k*^(*t*), and its expression is shown in the following formula:

(11) $$\begin{array}{c} p_{ij}^{k}t=\left\{\begin{array}{c} \frac{{\left[p_{ij}^{k}t\right]}^{\alpha }{\left[\eta_{ij}t\right]}^{\beta }}{\sum_{s=allowed_{k}}{\left[p_{ij}^{k}t\right]}^{\alpha }{\left[\eta_{ij}t\right]}^{\beta }},if\;j\in allowed_{k};\\ 0,\;or\;other \end{array}\right.. \end{array}$$

The residual information factor is *α*, the heuristic information factor is *β*, and the set of ant feasible paths is *allowed*_*k*_, as shown in the following formula:

(12) $$\begin{array}{c} allowed_{k}\in \left\{X_{s}|d_{sj}\leq r,s=1,2,\ldots ,N\right\}. \end{array}$$

The heuristic function is expressed as *η*_*ij*_(*t*), and its formula is as follows:

(13) $$\begin{array}{c} \eta_{ij}t=\frac{r}{d_{ij}}=\frac{r}{\sqrt{\sum_{k=1}^{m}p_{k}{\left(X_{ik}-C_{jk}\right)}^{2}}}. \end{array}$$

As can be seen from formula (13), the heuristic function increases with the increase of cluster radius, that is, the probability of selecting the corresponding cluster center increases. In addition, the heuristic function decreases with the increase of the distance between the pixel and the cluster center, that is, the probability of ant individuals selecting the corresponding cluster for merging decreases.

The main judgment basis for whether a pixel belongs to a cluster center is shown in the following formula:

(14) $$\begin{array}{c} p_{ij}^{k}\left(t\right)>p_{0}. \end{array}$$

If formula (14) is not met, the pixels are not merged into the cluster.

After one iteration, all ants need to update the cluster center and intraclass dissimilarity. As shown in formulas (15) and (16), it is a new calculation method of cluster center and dissimilarity.

(15) $$\begin{array}{c} {\tilde{C}}_{j}=\frac{1}{j}\sum_{k=0}^{j}\left(x_{k}\right), \end{array}$$

where *k* ∈ (1,2,…, *j*); the new cluster center is expressed as ${\tilde{C}}_{j}$.

(16) $$\begin{array}{c} \tilde{\varepsilon }=\sum_{j=1}^{k}\sum_{k=1}^{j}\sqrt{\sum_{i=1}^{m}{\left(X_{ki}-C_{ji}\right)}^{2}}. \end{array}$$

The new dissimilarity is expressed as $\tilde{\varepsilon }$.

## 4. Experimental Results of the Influence of Martial Arts on Spine Shape and Structure Based on Optimized Ant Colony Algorithm

In order to better test the improved CT image segmentation method based on the optimized ant colony algorithm, the segmentation time and iteration times are compared with the traditional fuzzy c-means classification method. First, the fuzzy rules are determined. Enter the corresponding parameters and activate some fuzzy rules. Only the rules whose membership degree is not 0 can be activated. The conclusion is obtained by comparing the membership degree, but the conclusion is not certain at this time. Finally, the conclusion is used to determine the actual output as shown in Figure 4.

It can be seen from the results in the figure that the time and iteration times of the two image segmentation methods increase with the increase of the number of clusters. Compared with the traditional fuzzy c-means classification method, the improved CT image segmentation method based on optimized ant colony algorithm is less sensitive to the number of clusters, and the increase of time and algorithm iteration is much less than the traditional fuzzy c-means classification algorithm. This shows that the improved CT image segmentation method based on optimized ant colony algorithm effectively overcomes the sensitivity of traditional methods to the number of clusters, improves the quality and efficiency of segmentation, and can provide more accurate information for the study of the impact of Wushu on the morphological structure of spine.

Huatuo Wuqinxi is an integral part of Chinese martial arts qigong, and it is also one of the national intangible heritages in Chinese traditional sports culture. The long-term development of Huatuo Wuqinxi is mainly because its movements are simple and easy to learn, suitable for all ages, and have a good mass foundation. Compared with other martial arts content, it can be more accepted and recognized by people. In this paper, 45 students with abnormal spinal morphology and structure in a primary school were selected as the experimental objects and randomly assigned to the experimental group and the control group. In the experimental group, eight subjects were patients with abnormal trunk inclination, fifteen subjects were patients with abnormal kyphosis angle, and two of them were patients with abnormal two conditions at the same time. In the control group, eight subjects had abnormal trunk inclination, fourteen subjects had abnormal kyphosis angle, and one of the subjects had abnormal two conditions at the same time.

Figure 5 shows the comparison of trunk tilt angle measurement results of experimental subjects before and after the experiment between experimental group and control group. Before the experiment, there was no significant difference in trunk tilt angle between the experimental group and the control group, while after the experiment, there was no significant change in trunk tilt angle between the two groups, *P* > 0.05, that is, there was no significant difference. The comparison *P* < 0.01 between the experimental group before and after the intervention shows that the trunk tilt angle of the experimental group is better than that before the intervention of Wuqinxi, and there is a significant difference.

As shown in Figure 6, the results of kyphosis angle of subjects in the experimental group and the control group before and after the experiment are compared. It can be seen from the figure that before the intervention of Wuqinxi, there was no obvious difference in the kyphosis angle between the experimental group and the control group, that is, *P* > 0.05, while after the intervention of Wuqinxi, the kyphosis angle of the experimental group was significantly improved, forming a very obvious difference with the control group. The kyphosis angle of the experimental group was significantly improved than that before the intervention of Wuqinxi, and there was significant difference between the two.

As shown in Figure 7, the comparison of spinal activity measurement results of subjects in the experimental group and the control group is shown. It can be seen from the figure that there is no significant difference in spinal activity between the experimental group and the control group before the intervention of Wuqinxi. After the intervention of Wuqinxi, the cervical spine activity and thoracic spine activity of the experimental group were better than those of the control group. There was no significant difference in lumbar spine activity between the experimental group and the control group. In addition, compared with before the intervention of Wuqinxi, the subjects in the experimental group improved their mobility in three directions: coronal, sagittal, and horizontal. The angle of motion of thoracic vertebrae was significantly improved in coronal and horizontal directions, and there were significant differences. The improvement of lumbar mobility in three directions is different, among which the improvement of lumbar mobility in sagittal plane is the most obvious and effective, with very significant difference. Second, there is a certain improvement in the activity of coronal plane, with significant difference. Finally, the activity of lumbar spine in the horizontal plane has a certain improvement trend, but there is no obvious difference.

Figure 8 shows the comparison of body balance results between the experimental group and the control group. It can be seen from the figure that before the intervention experiment of Wuqinxi, there was no significant difference in body balance between the two groups. After the intervention of Wuqinxi, there was a very significant difference between the experimental group and the control group. The measurement results of the experimental group were better than those of the control group. At the same time, the shoulder horizontal line of the experimental group was significantly improved compared with that before the intervention of Wuqinxi and showed a very obvious difference, namely, *P* < 0.01. The horizontal line of the posterior sacroiliac spine of the experimental group was also improved compared with the previous, with obvious differences.

In conclusion, the intervention of Huatuo Wuqinxi martial arts can improve the abnormal trunk tilt angle, kyphosis angle, and body balance angle of teenagers, and the effect is good. At the same time, Huatuo Wuqinxi can also improve the activity of teenagers' cervical spine and thoracic spine, showing obvious differences. There is also a certain improvement effect on the lumbar mobility. The improvement of the lumbar mobility in three aspects is different. The lumbar mobility is improved in the coronal plane and sagittal plane, showing a significant difference, but the improvement effect on the lumbar mobility in the horizontal plane is not obvious. Therefore, Huatuo Wuqinxi can improve the health status of teenagers' spine and improve the abnormal development of spine morphology and structure.

## 5. Conclusion

Adolescence and childhood are not only the golden periods for the development of human spine morphology and structure but also the key period for the physical development of adolescents and children. Therefore, adolescents' and children's spines are prone to abnormal development due to internal and external environment. At the same time, the bad living habits and learning pressure of teenagers have caused a certain pressure on the developing spine, which promotes its abnormal development. Most teenagers have slight spinal dysplasia such as chest hump and back compression, which can be improved through exercise intervention. In Chinese traditional sports culture, Wuqinxi is one of the national intangible cultural heritages, which has always had good results in health preservation. Therefore, this paper puts forward the research on the influence of martial arts on the spinal morphological structure based on the optimized ant colony algorithm. By optimizing the ant colony algorithm, we can improve the segmentation method of spinal CT image, improve the quality and efficiency of image segmentation, and provide more effective information and data for the later analysis of spinal morphological structure. Experiments show that compared with the traditional fuzzy c-means classification method, the improved CT image segmentation method based on optimized ant colony algorithm solves the problem of being sensitive to the number of clusters and improves the segmentation efficiency while ensuring the image segmentation quality. The comparison of the experimental results between the experimental group and the control group shows that the intervention of Wuqinxi Wushu can improve the abnormal trunk tilt angle and kyphosis angle of teenagers and achieve better results. In terms of adolescent spinal mobility, Wuqinxi has a good effect on the mobility of cervical spine and thoracic spine in three directions and has a significant effect on the mobility of lumbar spine in coronal plane and sagittal plane, but it has no obvious improvement on the mobility of lumbar spine in horizontal plane. Therefore, Huatuo Wuqinxi Wushu can improve the abnormal development of teenagers' spine and help teenagers improve their overall health. However, the study still has some limitations. The number of subjects is too small, so whether it can improve the health of adolescent spine is still controversial. Whether it is representative to improve the abnormal development of spinal morphology and structure remains to be discussed.

## Figures and Tables

**Figure 1:** Comprehensive view of spine.

**Figure 2:** Schematic diagram of ant colony foraging behavior in natural biosphere.

**Figure 3:** Improved CT image segmentation flowchart with optimized ant colony algorithm.

**Figure 4:** The traditional fuzzy c-means classification method is based on the improved CT image segmentation method of optimized ant colony algorithm.

**Figure 5:** Comparison of trunk tilt angle measurement results between experimental group and control group before and after experiment.

**Figure 6:** Comparison of kyphosis angle between experimental group and control group before and after experiment.

**Figure 7:** Comparison of measurement results of spinal mobility between experimental group and control group.

**Figure 8:** Comparison of body balance results between experimental group and control group.

## Data Availability

The data used to support the findings of this study are available from the corresponding author upon request.
